The article "Clinical Factors of Blood Transfusion-Related Acute Lung Injury and Changes in Levels of Treg-Related Cytokines" was retracted in 2024. Reasons: signs of a paper mill; suspected computer-generated content; unreliable results or conclusions; concerns about the data.

# Clinical Factors of Blood Transfusion-Related Acute Lung Injury and Changes in Levels of Treg-Related Cytokines

**DOI:** 10.1155/2022/7344375

**Published:** 2022-05-27

**Authors:** Lifang Sun, Yu Liu

**Affiliations:** ^1^Department of Blood Transfusion, Tianshui First People's Hospital, Tianshui, Gansu 741000, China; ^2^Department of Laboratory, Tianshui First People's Hospital, Tianshui, Gansu 741000, China

## Abstract

**Objective:**

Analysis of clinical factors and changes in regulatory T cell (Treg)-related cytokine levels in transfusion-associated acute lung injury (TRALI).

**Methods:**

62 patients who underwent blood transfusion and developed TRALI (TRALI group) in our hospital between January 2018 and December 2021 and 58 patients who did not develop TRALI (non-TRALI group) from blood transfusion were selected to collect clinical data from patients and construct a logistic regression model to analyze clinical risk factors for TRALI. Based on the prognosis of TRALI patients, they were divided into survival group (50 cases) and death group (12 cases), and serum CD4 + CD25 + Treg and Treg-related cytokines (interleukin 10 (IL-10), transforming growth factor-*β* (TGF-*β*)) levels were compared between the two groups, and the correlation between CD4 + CD25 + Treg and IL-10 and TGF-*β* was analyzed by Pearson.

**Results:**

The differences in smoking history, human leukocyte antigen (HLA) antibody II, pretransfusion shock, and CD4 + CD25 + Treg between the TRALI group and non-TRALI group were statistically significant (*P* < 0.05). Logistic regression analysis showed that HLA antibody II and increased CD4 + CD25 + Treg were independent risk factors of TRALI (*P* < 0.05). The levels of CD4 + CD25 + Treg, IL-10, and TGF-*β* in the death group were significantly higher than those in the survival group (*P* < 0.05). CD4 + CD25 + Treg was positively correlated with levels of IL-10 and TGF-*β* (*P* < 0.05).

**Conclusion:**

Elevated HLA antibody II and CD4 + CD25 + Treg are the main clinical risk factors for TRALI, and CD4 + CD25 + Treg may be involved in immunosuppression by increasing the expression levels of IL-10 and TGF-*β*. Early clinical monitoring of changes in Treg-related cytokine levels can provide some guidance for prognostic assessment of TRALI patients.

## 1. Introduction

Transfusion-related acute lung injury (TRALI) is an acute lung injury that occurs during or within 6 h after the completion of a transfusion and is characterized by hypoxemia, noncardiogenic pulmonary edema, and sudden onset of respiratory distress, with a poor prognosis. Studies have shown that TRALI has the highest mortality rate among transfusion reactions; however, the specific pathophysiological mechanisms are not fully understood and the diagnosis and treatment are challenging [1, 2]. At present, epidemiological data on TRALI are mainly obtained through active reporting by medical institutions, and fewer clinical case reports and basic studies are available, probably due to the lack of awareness of this adverse reaction among front-line clinical physicians and unstandardized diagnostic criteria, resulting in a relatively excessive rate of clinical misdiagnosis or underdiagnosis [3, 4]. TRALI is fast-onset, difficult to identify, and some patients are at a higher risk of developing TRALI, and it has been previously reported that critical patients are at a higher risk of developing TRALI, so timely detection and effective management in the clinic is important to improve their prognosis, and understanding the factors affecting TRALI can provide important guidance for its clinical management [5, 6].

At present, the specific pathogenesis of TRALI has not been fully clarified in clinical practice, and previous studies have pointed to the presence of immunosuppression in the early stages of TRALI development [7]. Regulatory T cells (Treg) belong to a subset of T cells that perform regulatory functions, and one of the better understood natural Treg is CD4 + CD25 + Treg. Relevant studies have shown that CD4 + CD25 + Treg can negatively regulate immunity through its related cytokines, effectively inhibit T cells, which are the main cells that maintain peripheral immune tolerance [8]. At this stage, domestic research on TRALI is mainly in the form of a review, and there are few reports on the influencing factors of TRALI and Treg cytokines. Based on this, this paper analyzed the clinical factors of TRALI and the changes of Treg-related cytokine levels, hoping to provide guidance for clinical practice.

## 2. Materials and Methods

### 2.1. General Information

62 patients who underwent blood transfusion and developed TRALI (TRALI group) in our hospital between January 2018 and December 2021 and 58 patients who did not develop TRALI (non-TRALI group) from blood transfusion were selected. The inclusion criteria are as follows: (1) TRALI patients met the relevant diagnostic criteria for TRALI [9]; (2) first diagnosis; (3) no recent history of immunosuppressive therapy; (4) complete clinical data; (5) symptoms occurred during the transfusion of blood or (and) blood products, or within 6 h after the transfusion of blood and/or blood products. The exclusion criteria are as follows: (1) combined trauma, rheumatoid arthritis, diabetes, central nervous system disease or infection, etc.; (2) cardiogenic pulmonary edema and sepsis caused by transfusion of contaminated blood products, etc.; (3) cancer patients; (4) lung injury caused by other reasons; (5) respiratory insufficiency was present before the transfusion.

### 2.2. Methods

The clinical data of patients were collected, including gender, age, body mass index (BMI), smoking history, surgical history, perioperative blood transfusion volume, total infusion volume, human leukocyte antigen (HLA) antibody I, and HLA antibody II, whether they were in shock before transfusion, whether they were treated with mechanical ventilation, and whether they had combined liver disease.

Peripheral venous blood samples were drawn from patients, and 50 *μ*L of peripheral blood mononuclear cells (PBMCs) were separated according to Ficoll density gradient centrifugation. 10% fetal bovine serum (50 mL of control) was added to resuspend the cells, and a flow cytometer (model: BD FACSCalibur) was taken for the CD4 + CD25 + Treg assay. Another PBMC suspension was taken, the supernatant was separated by centrifugation for 10 min (controlled at 1500 r/min), and then the levels of interleukin 10 (IL-10) and transforming growth factor-*β* (TGF-*β*) were measured by the enzyme-linked immunosorbent assay. The relevant test kits were purchased from Shuangyin Biotechnology Co.

The prognosis of TRALI patients during hospitalization was recorded and divided into the survival group and death group.

### 2.3. Statistical Processing

The SPSS 20.0 software was used for data analysis, the count data were expressed as “n and (%),” and the *χ*^2^ test was used; the measurement data that obeyed normal distribution were expressed as ($\bar{x}\pm s$), and the independent samples *t*-test was used between groups; logistic regression analysis was used for clinical factor analysis of TRALI; Pearson analysis was used for correlation analysis. *P* < 0.05 was considered statistically significant.

## 3. Results

### 3.1. Comparison of Clinical Data between TRALI Group and Non-TRALI Group

There was no statistical significance between the TRALI group and non-TRALI group in terms of their gender, age, BMI, surgical history, perioperative blood transfusion volume, total infusion volume, HLA antibody I, mechanical ventilation, combined liver disease, IL-10, and the levels of TGF-*β* (*P* > 0.05); the comparison was statistically significant in the following aspects: the smoking history, HLA antibody II, pretransfusion shock, CD4 + CD25 + Treg between the two groups (*P* < 0.05), as shown in Table 1.

### 3.2. Logistic Regression Analysis of Influencing Factors of TRALI

The independent variables were the indicators with statistical significance in the above analysis, and the specific assignments were shown in Table 2. Logistic regression analysis showed that elevated HLA antibody II and CD4 + CD25 + Treg were independent clinical risk factors for TRALI (*P* < 0.05), as shown in Tables 2 and 3.

### 3.3. Comparison of the Levels of CD4 + CD25 + Treg, IL-10, and TGF-*β* between Survival Group and Death Group

The levels of CD4 + CD25 + Treg, IL-10, and TGF-*β* in the death group were significantly higher than those in the survival group (*P* < 0.05), as shown in Table 4 and Figures 1∼ and 3.

### 3.4. Correlation Analysis

CD4 + CD25 + Treg in TRALI patients was positively correlated with the levels of IL-10 and TGF-*β* (*r* = 0.647, 0.574, both *P* < 0.001), as shown in Figures 4 and 5.

## 4. Discussion

Previous studies have shown that smoking history and pretransfusion shock can increase the risk of TRALI [10]. This study showed that the proportion of patients with smoking history and pretransfusion shock in the TRALI group was significantly higher than that in the non-TRALI group, indicating that smoking history and pretransfusion shock may affect the production of TRALI. Cigarettes contain a large amount of oxidant substances and smoking can affect the oxidative antioxidant balance in the lung. Glutathione (GSH) is the main antioxidant in the lung and plays an important defense role in the corresponding oxidant-mediated inflammatory response and lung injury, and smoking can inhibit GSH [11, 12]. Sympathetic excitation of the body after hemorrhagic shock promotes the secretion of catecholamines, leukotrienes, angiotensin, and endothelin by the renin-angiotensin system (RAS), while the coagulation-fibrinolytic system is also activated, all of which promote pulmonary vasoconstriction, causing a decrease in pulmonary blood flow and affecting capillary permeability, leading to ischemia-reperfusion injury in the lungs [13, 14]. However, this study found that smoking history and pretransfusion shock were not independent risk factors for TRALI, which may be related to the small sample size of this study, which may have a certain impact on the stability of the logistic model, and it is easier to obtain negative results.

During blood transfusion therapy, the perfusion products contain anti-leukocyte antibodies derived from the blood donor, which are associated with TRALI, such as anti-neutrophil antibodies with related homologs, anti-leukocyte antibodies type 1 as well as type 2, but not all antibodies are associated with an increased incidence of TRALI [15]. This study found that HLA antibody II was an independent clinical risk factor for TRALI. Reasons for this may be that HLA antibodies can bind to antigens distributed on the surface of neutrophils (NEUT), which allows a significant activation of NEUT and damage to endothelial cells of lung tissue, thus increasing the risk of TRALI. Previous studies have shown that within the blood donor population, HLA antibodies are present in about 10% of pregnant women, with a 3- to 4-fold increase in this percentage in those with at least three pregnancies [16]. Therefore, strict differentiation of donor blood is recommended, and TRALI mediated by plasma products can be avoided by excluding pregnant women. CD4 + CD25 + Treg can play a dedicated immunosuppressive role by expressing the production of CD4+ and CD25+ and promoting the formation of transcription factor Foxp3 to play an immunosuppressive function, participating in the drift of T cells to helper T cells 2 (Th2), and effectively regulating Th1/Th2 balance state and induce immune tolerance [17, 18]. After multivariate analysis, this study showed that the increased level of CD4 + CD25 + Treg was a clinical risk factor for TRALI. According to the “double-whammy theory,” the human body will experience an excessive inflammatory response when stimulated by events such as severe trauma, traumatic surgery, and massive blood loss, resulting in the activation of NEUT and the accumulation of NEUT in the lungs through the pulmonary circulatory system [19, 20]. When a large number of blood transfusions are given, the platelet fragments, related denatured protein molecules, and leukocytes as well as allogeneic immune components in blood products are more likely to react with immune components in the human circulatory system, increasing CD4 + CD25 + Treg and enhancing NEUT chemotaxis, making the pulmonary microcirculation disorder more serious, thus damaging alveolar epithelial cells and endothelial cells [21].

It has been reported [22] that Treg-related cytokines (IL-10 and TGF-*β*) show abnormal changes when the immune function of the body is disturbed. In this study, the levels of CD4 + CD25 + Treg, IL-10, and TGF-*β* in the death group were significantly higher than those in the survival group, indicating that patients with increased CD4 + CD25 + Treg and high expression of IL-10 and TGF-*β* had a higher prognosis. Correlation analysis showed that CD4 + CD25 + Treg was positively correlated with the levels of IL-10 and TGF-*β*, and CD4 + CD25 + Treg may affect the prognosis of TRALI patients by increasing the expression levels of IL-10 and TGF-*β*, which may be a new target for immune blockade in the body. The results suggest that CD4 + CD25 + Treg may be a new target for immune blockade and provide a basis for clinical efficacy and prognosis assessment of TRALI.

To sum up, the clinical risk factors of TRALI mainly include HLA antibody II, high CD4 + CD25 + Treg, etc. CD4 + CD25 + Treg may affect the prognosis of TRALI patients by upregulating the expression of IL-10 and TGF-*β*, and early monitoring of them is beneficial to the prognosis assessment of patients with TRALI.

## Figures and Tables

**Figure 1:** Distribution of CD4 + CD25 + Treg in survival group and death group.

**Figure 2:** Distribution of IL-10 in survival group and death group.

**Figure 3:** Distribution of TGF-*β* in survival group and death group.

**Figure 4:** Relationship between CD4 + CD25 + Treg and IL-10.

**Figure 5:** Relationship between CD4 + CD25 + Treg and TGF-*β*.

**Table 1:** Comparison of clinical data between TRALI group and non-TRALI group (n (%), $\bar{x}\pm s$).

Clinical data	TRALI group (*n* = 62)	Non-TRALI group (*n* = 58)	*χ* ^2^ or *t*	*P* value
Gender			0.595	0.441
Male	32 (51.61)	34 (58.62)		
Female	30 (48.39)	24 (41.38)		
Age (years)	49.56 ± 7.94	49.71 ± 7.90	0.587	0.558
BMI (kg/m^2^)	23.82 ± 2.15	23.52 ± 2.47	0.711	0.479
Smoking history			12.035	0.001
Yes	33 (53.23)	13 (22.41)		
No	29 (46.77)	45 (77.59)		
Surgical history			0.155	0.694
Yes	53 (85.48)	51 (87.93)		
No	9 (14.52)	7 (12.07)		
Perioperative blood transfusion volume (mL)	3747.24 ± 521.12	3590.63 ± 515.22	1.654	0.101
Total infusion volume (mL)	4222.49 ± 637.59	4228.76 ± 598.01	0.055	0.956
HLA antibody I			0.028	0.868
Yes	7 (11.29)	6 (10.34)		
No	55 (88.71)	52 (89.66)		
HLA antibody II			11.749	0.001
Yes	16 (25.81)	2 (3.45)		
No	46 (74.19)	56 (96.55)		
Pretransfusion shock			16.421	＜0.001
Yes	40 (64.52)	16 (27.59)		
No	22 (35.48)	42 (72.41)		
Mechanical ventilation			2.724	0.099
Yes	35 (56.45)	24 (41.38)		
No	27 (43.55)	34 (58.62)		
Combined liver disease			1.230	0.268
Yes	33 (53.23)	25 (43.10)		
No	29 (46.77)	33 (56.90)		
CD4 + CD25 + Treg (%)	38.39 ± 4.62	26.40 ± 5.37	13.137	＜0.001
IL-10 (ng/L)	35.79 ± 5.65	34.84 ± 5.85	0.905	0.367
TGF-*β* (*μ*g/L)	49.62 ± 8.19	48.93 ± 7.78	0.472	0.638

**Table 2:** Variable assignment.

Variable	Assignment
Y : TRALI	0 : non-TRALI
	1 : TRALI

X1 : smoking history	0 : no
	1 : yes

X2 : HLA antibody II	0 : no
	1 : yes

X3 : pretransfusion shock	0 : no
	1 : yes

X4 : CD4 + CD25 + Treg	Enter the value directly

**Table 3:** Logistic regression analysis.

Factor	*β*	SE	Wald value	OR value	95% CI	*P* value
Smoking history	−0.664	1.753	0.144	0.515	0.017～15.989	0.705
HLA antibody II	4.729	1.694	7.788	113.182	4.091～3131.414	0.005
Pretransfusion shock	0.907	1.650	0.302	2.477	0.098～62.866	0.582
CD4 + CD25 + Treg	0.574	0.114	25.274	1.775	1.420～2.220	＜0.001
Constant	−19.586	3.901	25.207	＜0.001	—	＜0.001

**Table 4:** Comparison of the levels of CD4 + CD25 + Treg, IL-10, and TGF-*β* between survival group and death group ($\bar{x}\pm s$).

Group	CD4 + CD25 + Treg (%)	IL-10 (ng/L)	TGF-*β* (*μ*g/L)
Survival group (*n* = 50)	37.76 ± 4.55	34.92 ± 5.05	48.09 ± 7.20
Death group (*n* = 12)	41.00 ± 4.14	39.39 ± 6.75	56.01 ± 9.27
*t*	2.251	2.574	3.233
*P* value	0.028	0.013	0.002

## Data Availability

The data used and analyzed during the current study are available from the corresponding author.

## References

[1] Baudel J. L., Vigneron C., Pras-Landre V. (2020). Transfusion-related acute lung injury (TRALI) after intravenous immunoglobulins: French multicentre study and literature review. *Clinical Rheumatology*.

[2] Hu A., Chen W., Wu S. (2020). An animal model of transfusion‐related acute lung injury and the role of soluble CD40 ligand. *Vox Sanguinis*.

[3] Vlaar A. P. J., Kleinman S. (2020). An update of the transfusion-related acute lung injury (TRALI): a proposed modified definition and classification scheme definition. *Indian Journal of Hematology and Blood Transfusion*.

[4] Gregory Rivera M., Sampson A. C., Hair P. S. (2020). Incompatible erythrocyte transfusion with lipopolysaccharide induces acute lung injury in a novel rat model. *PLoS One*.

[5] Hu L., Wang B., Jiang Y. (2021). Risk factors for transfusion-related acute lung injury. *Respiratory Care*.

[6] Vlaar A. P. J., Toy P., Fung M. (2019). A consensus redefinition of transfusion‐related acute lung injury. *Transfusion*.

[7] McVey M. J., Kapur R., Cserti-Gazdewich C., Semple J. W., Karkouti K., Kuebler W. M. (2019). Transfusion-related acute lung injury in the perioperative patient. *Anesthesiology*.

[8] Liu Y., Li C., Yang Y. (2021). The TGF‐*β*/miR‐31/CEACAM1‐S axis inhibits CD4 + CD25 + Treg differentiation in systemic lupus erythematosus. *Immunology & Cell Biology*.

[9] Toy P., Popovsky M. A., Abraham E. (2005). Transfusion-related acute lung injury: definition and review. *Critical Care Medicine*.

[10] McVey M. J., Weidenfeld S., Maishan M. (2021). Platelet extracellular vesicles mediate transfusion-related acute lung injury by imbalancing the sphingolipid rheostat. *Blood*.

[11] Dawod Y. T., Cook N. E., Graham W. B., Madhani-Lovely F., Thao C. (2020). Smoking-associated interstitial lung disease: update and review. *Expert Review of Respiratory Medicine*.

[12] Kalinina E., Novichkova M. (2021). Glutathione in protein redox modulation through S-glutathionylation and S-nitrosylation. *Molecules*.

[13] Preuss J. M., Burret U., Gröger M. (2021). Impaired glucocorticoid receptor signaling aggravates lung injury after hemorrhagic shock. *Cells*.

[14] Zhang L., Wang W., Qiao Q. Q. (2019). Pré‐condicionamento com dexmedetomidina protege contra lesão pulmonar em ratos com choque hemorrágico. *Brazilian Journal of Anesthesiology*.

[15] Jug R., Anani W., Callum J. (2021). A possible case of recipient anti‐neutrophil and anti‐human leukocyte antigen antibody‐mediated fatal reverse transfusion‐related acute lung injury. *Transfusion*.

[16] Belizaire R., Mack J., Kadauke S., Kim Y., Saidman S., Makar R. S. (2019). Red blood cell alloantibodies are associated with increased alloimmunization against human leukocyte antigens. *Transfusion*.

[17] Wang R., Huang K. (2020). CCL11 increases the proportion of CD4+CD25+Foxp3+ Treg cells and the production of IL-2 and TGF-*β* by CD4+ T cells via the STAT5 signaling pathway. *Molecular Medicine Reports*.

[18] Mao Q.-F., Shang-Guan Z.-F., Chen H.-L., Huang K. (2019). Immunoregulatory role of IL-2/STAT5/CD4+CD25+Foxp3 Treg pathway in the pathogenesis of chronic osteomyelitis. *Annals of Translational Medicine*.

[19] Akimova T., Zhang T., Christensen L. M. (2021). Obesity-related IL-18 impairs T-regulatory cell function and promotes lung ischemia-reperfusion injury. *American Journal of Respiratory and Critical Care Medicine*.

[20] Roubinian N. H., Triulzi D. J. (2019). Transfusion-associated circulatory overload and transfusion-related acute lung injury. *Hematology-Oncology Clinics of North America*.

[21] Song J., Gong Y.-H., Yan X. (2021). Regulatory T cells accelerate the repair process of renal fibrosis by regulating mononuclear macrophages. *The American Journal of the Medical Sciences*.

[22] da Silva Alves R., Abdalla D. R., Iunes D. H. (2020). Influence of an exergaming training program on reducing the expression of IL-10 and TGF-*β* in cancer patients. *Games for Health Journal*.

